# Detection and phylogeny of *Staphylococcus aureus* sequence type 398 in Taiwan

**DOI:** 10.1186/s12929-019-0608-8

**Published:** 2020-01-03

**Authors:** Yhu-Chering Huang, Chih-Jung Chen

**Affiliations:** 1 Division of Pediatric Infectious Diseases, Chang Gung Memorial Hospital, Taoyuan, Taiwan; 2 Chang Gung University College of Medicine, Taoyuan, Taiwan; 3 Department of Pediatrics, Chang Gung Memorial Hospital, No. 5, Fu-Shin Street, Gueishan, 333 Taoyuan, Taiwan

**Keywords:** Methicillin-resistant *Staphylococcus aureus*, Sequence type 398, Pulsotype, Taiwan

## Abstract

**Background:**

Methicillin-resistant *Staphylococcus aureus* (MRSA) ST398 is a livestock associated-bacterium that is most prevalent in Europe. Human-adapted MRSA ST398 was recently reported from China, but there is no data available yet for Taiwan.

**Methods:**

To identify *S. aureus* ST398 isolates, we examined 6413 *S. aureus* isolates (5632 MRSA and 781 susceptible strains) that were collected in Taiwan between 1995 and 2017. If isolates could not be typed by pulsed-field gel electrophoresis upon *Sma* I digestion, we performed further characterization and complete genome sequencing.

**Results:**

We identified 18 ST398 *S. aureus* isolates from 16 subjects (0.28%), including 6 sensitive and 12 resistant strains. Of these, 14 were colonizing isolates, 3 were clinical (infecting) isolates and one isolate was from a pork specimen. All 3 infecting isolates were MSSA strains identified in 2015 from two children with recurrent otitis media or sinusitis. The other 3 MSSA isolates were identified from workers handling pork (2) or pork meat (1) in 2015. The first 5 MRSA colonizing isolates were identified from residents in two nursing homes in 2012. Six MRSA isolates were identified from residents and foreign employees at a nursing home in 2016 and one MRSA from a foreign worker in 2017. Phylogenetic analysis of genome sequences indicated that all 12 local ST398 MRSA strains cluster together, human-adapted and phylogenetically related to a human MRSA strain identified in China in 2002. Two local MSSA isolates could be linked to isolates from livestock. The toxin profiles were similar for the MRSA and MSSA isolates.

**Conclusions:**

Our results demonstrate that *S. aureus* ST398 was present in Taiwan in 2012 and potentially earlier. Although some isolates could be linked to livestock, most ST398 *S. aureus* isolates identified in Taiwan, particularly MRSA, represent human-adapted strains. Local transmission of human-adapted MRSA ST398 strains has occurred in nursing homes in Taiwan, possibly after import from China. Further surveillance is needed.

## Introduction

In addition to being a human pathogen, methicillin-resistant *Staphylococcus aureus* (MRSA) can also colonize and cause diseases in a variety of animals, which as known as livestock-associated MRSA (LA-MRSA) [1, 2]. In the past decade, LA-MRSA has been increasingly identified in humans and has been associated with very severe diseases and even death [1, 2]. MRSA sequence type (ST) 398 was the first identified LA-MRSA [1–4], initially identified in Europe and subsequently identified in areas outside Europe, including Asian countries, such as South Korea [5, 6], Singapore [7], Japan [8–10] and Thailand [11]. Lately, human-adapted ST398 community-associated (CA) MRSA, evolving from methicillin-susceptible *S. aureus* (MSSA) demonstrated by whole genome sequencing analysis, was reported from China [12–14] and caused severe human disease and even death. Human-adapted MRSA is genetically different from LA-MRSA [12, 13] and is associated with absence of the *tet*M resistance determinant and presence of a variant of prophage 3, containing the immune evasion complex (IEC) genes encoding the chemotaxis inhibitory protein (*chp*), staphylococcal complement inhibitor (*scn*), and staphylokinase (*sak*).

In Taiwan, MRSA was first documented in early 1980s and rapidly increased in 1990s [15]. In contrast to a declining trend of HA-MRSA incidence observed in 2000s, CA-MRSA infections have been increasingly reported, particularly in pediatric patients [15–17]. LA-MRSA was also identified from pigs and humans recently and caused minor to life-threatening human infections [18]. Most LA-MRSA in Taiwan belonged to ST9 while ST398 was not specifically reported yet [15–18]. Recently, we identified five MRSA ST398 isolates in a survey for MRSA carriage in nursing homes in 2012 [19], prompting our study on this strain in Taiwan to figure out the perspective of MRSA ST398 in Taiwan. Herein, we report the detection, and phylogenetic analysis of ST 398 *S. aurues* isolates identified in our laboratory in Taiwan as well as the epidemiologic information of these isolates.

## Methods

For surveillance of molecular epidemiology of *S. aureus*, we collected and molecularly characterized (at least by pulsed-field gel electrophoresis (PFGE)) a total of 6413 *S. aureus* isolates (MRSA, 5632 and MSSA, 781) island-wide in Taiwan between 1995 and 2017 in our laboratory, which is located at Chang Gung Memorial Hospital (CGMH). Identification of *Staphylococcus aureus* was confirmed by the conventional methods according to Clinical and Laboratory Standards Institute (CLSI) guidelines [20]. MRSA was screened by cefoxitin disc first and confirmed by the detection of *mec*A gene. The distribution of these MSSA and MRSA isolates stratified by identified years and sources is shown in Table 1. In addition to CGMH, the isolates were also collected from at least 10 hospitals in Taiwan. Of 105 non-human MRSA isolates, 93 isolates were from pigs, 9 from the environmental objects, 2 from the bus and one from the pork. Of 15 non-human MSSA isolates, 10 isolates were from the bus and 5 from the pork. The clinical (infecting) isolates were identified from any body site, and by epidemiologic criteria, around 460 isolates were community-associated (without risk factors for MRSA acquisition) while - than 90% of the remaining 2592 isolates were estimated to be healthcare-associated. Among the 2580 MRSA colonizing isolates, 1632 isolates (63%) were identified from children < 18 years of age, including infants hospitalized in neonatal intensive care units (NICUs), neonates in nurseries, children for well baby clinic visits, school children and case patients, while 838 isolates were from adult patients, parturient mothers and elderly stayed in nursing homes. Forty-five percent of the 2580 MRSA colonizing isolates were identified from the subjects without risk factors for MRSA acquisition.

**Table 1:** Distribution of methicillin-resistant *Staphylococcus aureus* and methicillin-susceptible *Staphylococcus aureus* collected island-wide between 1995 and 2017 and molecularly characterized in Chang Gung Memorial Hospital, stratified by identified years and sources

Period/ population	MRSA No. (%)			MSSA No. (%)			Total No. (%)
	Clinical	Colonizing	Subtotal	Clinical	Colonizing	Subtotal	
1995–2004	1307	502	1809 (32)	51	0	51 (6.5)	1860 (29)
2005–2010	1102	1435	2537 (45)	6	311	317 (41)	2854 (45)
2011–2017	643	643	1286 (23)	190	223	413 (53)	1699 (26)
Total	3052 (54)	2580 (46)	5632	247 (32)	534 (68)	781	6413
Pediatric	980	1632	2612 (46)	184	218	402	3014 (47)
Adults	334	838	1172 (21)	12	301	313	1485 (23)
Unclassified	1738^a^	5	1743 (31)	51	0	51	1794 (28)
Non-human	0	105	105 (1.9)	0	15	15	120 (1.9)

^a^We estimated more than 90% of the isolates were from adult patients

### Identification and characterization of *S. aureus* ST398 isolates

Because ST398 *S. aureus* cannot be digested by *Sma*I on pulsed-field gel electrophoresis (PFGE), we first examined the isolates which could not be digested by *Sma*I to identify potentially ST398 *S. aureus* isolates. For those not typeable by *Sma*I digested PFGE, we performed multilocus sequence typing (MLST) to confirm the isolates to be ST398 or not. For ST398 *S. aureus* isolates, we performed further characterizations, including staphylococcal cassette chromosomal typing (SCC*mec*), *spa* typing, and detection of Panton-Valentine leukocidin (PVL) genes and some other toxin genes. All the methods were performed according to the procedures described elsewhere [19, 21, 22]. The antibiotic susceptibility test was performed on Mueller–Hinton agar with disk-diffusion method according to the CLSI guidelines [20] and included teicoplanin, linezolid, fusidic acid, trimethoprim/sulfamethoxazole, ciprofloxacin, doxycycline, erythromycin, clindamycin and penicillin. The susceptibility to vancomycin was determined by minimal inhibition concentration.

### Whole genome sequencing (WGS) and phylogenetic analysis

All the ST398 *S. aureus* isolates identified were subjected to whole genome sequencing (WGS), which was performed on an Illumina MiSeq sequencer (Illumina, San Diego, CA, USA) [23] and the results were deposited at DDBJ/ENA/GenBank under the accession PRJNA554199. The multi-alignment of the core genomes was conducted with the Mauve procedure and the multi-alignment file was subsequently used for maximum likelihood phylogeny construction of the ST398 strains based on the single nucleotide polymorphisms (SNPs) outside of the potential recombination regions with the gubbins procedure [24, 25]. The length of the alignment was 2,561,981 bp and the SNP numbers for the isolates are shown in Fig. 2. The resistance and the virulence genes carried by the local ST398 strains were detected by the srst2 software using the ARG-ANNOT database and VFDB (http://www.mgc.ac.cn/VFs), respectively [26, 27]. The final phylogenetic tree and the data of carried resistance and virulence genes were input into Interactive Tree Of Life (http://itol. embl.de) for further annotation.

To clarify the genetic relatedness of the strains in Taiwan and global isolates, 87 published whole genome sequences data of ST398 *S. aureus* strains were downloaded from the GenBank database and included for analysis. In addition to the maximum likelihood phylogeny construction mentioned above, the Bayesian analysis of the molecular sequences using Markov chain Monte Carlo was performed with the BEAST procedure (v 1.10.4) to estimate the time to most common recent ancestor [28]. A HKY model with estimated base frequencies, strict clock type and constant size of tree prior was used. Three independent chains were run for 100 million generations and sampling every 1000 generations. The effect sample size values were checked by tracer (v1.7.1) and were greater than 200. A burn-in of 10 million states was removed from each of the three independent runs before combining the results from those runs with the logcombiner program (v 1.10.4) from the BEAST package. The final tree was output with Figtree (https://github.com/rambaut/figtree/releases). The resistance and the virulence genes carried by the local ST398 strains were detected by the srst2 software using the ARG-ANNOT database and VFDB (http://www.mgc.ac.cn/VFs/.), respectively [26, 27].

Clinical features and sources of the ST398 *S. aurues* isolates were retrospectively reviewed. This study was approved by Chang Gung Medical Foundation Institutional Review Board (IRB No.:201600069B0).

## Results

### Identifying ST398 *S. aureus* isolates in Taiwan

Among the pool of 6413 isolates, we identified 18 (0.28%) ST398 *S. aureus* isolates, including 12 MRSA and 6 MSSA. Only three MSSA isolates from two patients were clinical isolates, 14 isolates were colonizing isolates and one isolate was from the pork meat (non-human isolate. Both patients with infecting isolates were children; one 4-year-old girl (subject 10) had combined immunodeficiency and presented with recurrent otitis media; the other patient, a 2-year-old boy, manifested as sinusitis. Among the three colonizing MSSA isolates, two MSSA isolates were identified from two workers handling pork (one worked in a traditional wet market and the other worked in a supermarket), and one MSSA isolate from the pork meat in a supermarket. All 6 MSSA isolates were identified in 2015.

All of the 12 MRSA were colonizing isolates. Five MRSA isolates were identified from five residents in two nursing homes (NHs) in a survey conducted in 2012 for MRSA carriage among residents and health care workers (HCWs) in 14 nursing homes island-wide [15]. Six MRSA isolates were identified from two residents (patient 11 had two isolates identified in 2 different surveys) and three foreign nursing workers (from the Philippines) in one nursing home in a longitudinal surveys (totally four surveys) conducted in 2016 for MRSA carriage among residents and HCWs in four NHs in northern Taiwan. The remaining one MRSA isolate was identified from a foreign worker recruited from Indonesia in 2017. The first ST398 MRSA isolate in Taiwan was identified in 2012 [15]. The detailed data of the 18 isolates are shown in Table 2.

**Table 2:** Detailed clinical features of the 16 subjects with 18 ST398 *Staphylococcus aureus* isolates identified in Taiwan

Strain name	Subject No.	Year of isolation	Age (years)	Status	Remarks
RR70	1	2012	69	Colonized	Survey in 14 nursing homes
RR69	2	2012	53	Colonized	Survey in 14 nursing homes
RR74	3	2012	63	Colonized	Survey in 14 nursing homes
RR82	4	2012	82	Colonized	Survey in 14 nursing homes
RR95	5	2012	72	Colonized	Survey in 14 nursing homes
AAS1^a^	6	2015	–	Non-human	Pork meat in a supermarket
AAS9^a^	7	2015	Unknown	Colonized	Survey for pork processing workers
ZS13^a^	8	2015	Unknown	Colonized	Survey for pork processing workers
OSSA1032^a^	9	2015	2	Sinusitis	Cured
OSSA1096^a^	10	2015	4	Otitis media	Combined immunodeficiency, Recurrent otitis
OSSA1105^a^	10	2015	4	Otitis media	Combined immunodeficiency, Recurrent otitis
ABR26	11	2016	86	Colonized (resident)	^b^Longitudinal survey in a nursing home (1st survey)
ABR171	11	2016	86	Colonized (resident)	(4th survey)
ABR112	12	2016	93	Colonized (resident)	(3rd survey)
ABR121	13	2016	29	Colonized (worker, Philippines)	(3rd survey)
ABR134	14	2016	30	Colonized (worker, Philippines)	(3rd survey)
ABR180	15	2016	26	Colonized (worker, Philippines)	(4th survey)
ACR49	16	2017	27	Colonized (worker, Indonesia)	Survey for foreign workers recruited to Taiwan

^a^these 6 isolates were methicillin-sensitive *Staphylococcus aureus*; others were MRSA

^b^the frequency of sampling in this longitudinal study was bi-monthly

### Molecular characteristics of ST398 *S. aureus* isolates in Taiwan

All 18 isolates were characterized as ST398 by MLST. All 12 MRSA isolates carried type V_T_ SCC*mec*, and belonged to *spa* type t034. The first five MRSA isolates identified in 2012 possessed PVL genes while the other seven isolates did not. The six MSSA isolates belonged to four *spa* types. Both MSSA isolates from patient 10 with recurrent acute otitis media belonged to *spa* type t1250, and both isolates from workers handling pork belonged to *spa* type t571.

All 18 isolates were susceptible to vancomycin, teicoplanin, linezolid, fusidic acid while 17 were susceptible to doxycycline, and trimethoprim/sulfamethoxazole. One MRSA (RR82) and MSSA (ZS13) isolate was resistant to ciprofloxacin. Of the six MSSA isolates, one isolate (ZS13) was non-susceptible to doxycycline, and four were resistant to penicillin (Table 3).

**Table 3:** Antibiograms^a^ of the 16 patients with 18 ST398 *Staphylococcus aureus* isolates identified in Taiwan

Strain name	Subject No.	CC	E	P	SXT	D	CIP
RR70	1	S	S	R	S	S	S
RR69	2	S	S	R	S	S	S
RR74	3	S	S	R	S	S	S
RR82	4	S	S	R	S	S	R
RR95	5	S	S	S	S	S	S
AAS1#	6	S	S	S	S	S	S
AAS9#	7	S	R	S	S	S	S
ZS13#	8	R	R	R	S	I	R
OSSA1032#	9	R	R	R	S	S	S
OSSA1096#	10	R	R	R	S	S	S
OSSA1105#	10	R	R	R	S	S	S
ABR26	11	S	S	R	S	S	S
ABR171	11	R	R	R	S	S	S
ABR112	12	R	R	R	I	S	S
ABR121	13	S	S	R	S	S	S
ABR134	14	S	S	R	S	S	S
ABR180	15	S	S	R	S	S	S
ACR49	16	S	S	R	S	S	S

*CC* clindamycin, *E* erythromycin, *P* penicillin, *SXT* trimethoprim-sulfamethoxazole, *D* doxycycline, *CIP* ciprofloxacin

^a^All 18 isolates were susceptible to vancomycin, teicoplanin, fusidic acid and linezolid

#These six isolates were methicillin-susceptible

### Whole genome sequencing and phylogenetic analysis of ST398 *S. aureus*

The core genome-based phylogeny of the 18 local strains and 87 global strains of ST398 is shown in Fig. 1a. Multiple likelihood analysis of SNPs in core genomes disclosed all twelve local ST398 MRSA strains were clustered together and were genetically related to a human MRSA strain (strain 36_CN_2002) isolated from China in 2002. The BEAST analysis (Fig. 1b) suggested that all of the ST398 MRSA human isolates from Taiwan shared the common ancestor in 1986 with a human strain (strain 36_CN_2002) isolated from China in 2002 and then were diverged in 2006. These findings suggested that the local ST398 MRSA shared the common ancestor of the isolate from China and had caused local transmission in some long-term care facilities in Taiwan after 2012. Of the six ST398 MSSA isolates, except for two strains (OSSA1096 and OSSA1105) isolated from the child with recurrent otitis media in different time points, the phylogeny of the local ST398 MSSA strains, though all of them were identified in the same year (2015), was very diverse. The number of SNPs between these MSSA isolates could be greater than 550, suggesting different origins of the isolates (Fig. 1a). The BEAST analysis suggested that all the ST398 MSSA isolates but the strain of ZS13 were derived from another ancestor in 1974, which was shared by some human isolates from France, United States and China between 2007 and 2009. The details of the comparative genomics of the ST398 strains were provided (Fig. 1).

**Fig. 1:** **a** Maximum likelihood phylogenetic analysis of 18 ST398 *Staphylococcus aureus* isolates from Taiwan based on single nucleotide polymorphisms in the core genomes. 87 global ST398 isolates were included for comparison. All 12 local ST398 human MRSA strains were clustered and were genetically related to a human MRSA strain (36_CN_2002) isolated from China in 2002. The phylogenetic tree was produced by gubbins procedure using the multi-alignment file of all ST398 genomes generated by Mauve procedure and finally annotated in the tree of life website (Methods for detailed description). **b** The estimated time to most common recent ancestor among the ST398 strains with the BEAST program. The phylogenetic tree of isolates from Taiwan and China were amplified for more clear display. All of the ST398 MRSA human isolates from Taiwan shared the most common recent ancestor in 1986 with the strain of 36_CN_2002 from China in 2002. All ST398 MSSA isolates but the strain of ZS13 shared the most common recent ancestor in 1974 with some isolates from France, United States and China identified between 2007 and 2009. Abbreviation: AT, Austria; BE, Belgium; CA, Canada; CH, Switzerland; CN, China; DE, Germany; DK, Denmark; ES, Spain; FI, Finland; FR, France; GF, French Guiana; HU, Hungary; IT, Italy; NL, The Netherlands; PE, Peru; PL, Poland; PT, Portugal; SI, Slovenia; TW, Taiwan; US, United States

The distributions of the virulence and resistance genes carried by these strains are displayed in Fig. 2. The resistant profile was distinct between MRSA and MSSA isolates while the toxin profile was relatively similar between both groups of the isolates. All 12 MRSA isolates were found to lack the tetM resistance gene and contain the immune evasion complex (IEC) genes, including chp, scn, and sak, which are genetic determinants previously associated with human origin and adaptation, thus suggesting a non-livestock-associated origin. All but 2 MSSA isolates (AAS1 and ZS13) were found to be human adapted. Strain ZS13, which was identified from a worker handling pork in a traditional wet market, had abundant resistant genes but was completely absent for the IEC genes, suggesting a livestock-associated MSSA isolate. Strain AAS1, identified from the pork specimen, had *sak* gene but absent for *tet*M determinant, *scn* gene and *chp* gene, implying a potential livestock-associated.

**Fig. 2:** The distributions of the virulence and resistance genes identified in the 18 ST398 *Staphylococcus aureus* isolates from Taiwan. Human-adapted immune evasion complex genes (*sak*, ch*p* and *scn* genes) were identified in all human ST398 isolates except Strain ZS13 but mostly missing in the isolate identified from the pork meat (strain AAS1). The figure was produced using the tree of life website (http://itol. embl.de)

## Discussion

To our knowledge, this is the first report focusing on MRSA ST398 in Taiwan. In this study, the first ST398 isolate was identified in 2012 from a resident in one nursing home in a survey conducted in 2012 for MRSA carriage [19], which suggests that ST398 existed in Taiwan since 2012 or earlier. Also, though the *S. aureus* isolates collected between 2012 and 2017 in our laboratory only accounted for 15.7% of the pool of 6413 *S. aureus* isolates which were collected between 1995 and 2017, all the 18 ST398 isolates in this study were identified since 2012, suggesting the identification increased markedly recently in Taiwan.

MRSA ST398 was first identified as a LA-MRSA and prevailed in Europe, then in the North America but rarely reported from Asian countries [1–4]. Human infections of LA-MRSA ST398 have been reported, particularly from Europe, since first identified from pigs [3, 4, 29–31] and may manifest from a minor infection of skin and soft tissue infection, to life-threatening events of necrotizing pneumonia, bloodstream infection and endocarditis, even resulting in subsequent lethality. LA-MRSA has become an important cause of skin and soft tissue infections (SSTIs) in previously healthy individuals in European countries with a low prevalence of MRSA [29, 30]. The strains can also cause several difficult-to-treat infections and even death in patients with or without exposure to livestock [32–34].

The prevalence of LA-MRSA among pigs in Asian countries varied widely by geographical locations [1, 2]. In most Asian countries, LA-MRSA isolates belong to ST9, but with different molecular characteristics [1, 2]. LA-MRSA ST9 was rarely reported to be associated with human diseases at present [35, 36]. In a lately report from Taiwan [18], LA-MRSA ST9 was identified in 0.24% of 3328 human MRSA clinical (infecting) isolates collected from 1998 to 2012 islandwide. However, LA-MRSA ST398 was rarely identified from Asian countries and only reported from Korea (in commercial pigs) [5, 6], Singapore (in experimental pigs in a hospital research) [7], Japan [8–10] and Thailand [11].

Human-adapted ST398 isolates, genetically different from LA clones, often cause life-threatening infections and share some genetic features for the adaptation to humans as hosts [12–14, 34]. Almost all previously reported human-adapted ST398 isolates are MSSA [12, 37]. Lately, eight cases, of which six were severe and two were fatal, infected with ST398 CA-MRSA without connection to livestock were reported from China [12]. Genomic analysis revealed that these highly infectious ST398 CA-MRSA isolates evolved from human-adapted methicillin-susceptible clones. Similar severe, even fatal, cases were also reported from Japan [8] and Australia [38]. This strain seemed to be spreading internationally and needs further surveillance and monitoring.

In this study, only three MSSA isolates from two children were infecting isolates and all three isolates were genetically human-adapted by WGS analysis, as reported from China [12, 37]. Both pediatric patients presented with respiratory tract infections, including acute otitis media and sinusitis. In contrast, all 12 MRSA ST398 isolates in the present study were colonizing isolates. No invasive diseases caused by these ST398 strains were identified yet in Taiwan.

In this study, toxin profiles showed that all 12 MRSA ST398 isolates and four of six MSSA ST398 isolates were human-adapted while only two MSSA ST398 isolates from a worker handling pork in a traditional wet market and a pork meat, respectively, were potentially livestock-associated, suggesting that LA-*S. aureus* ST398 isolates were still uncommonly circulating but potentially existed in Taiwan. Multiple likelihood analysis of SNPs in core genomes revealed that all twelve local ST398 MRSA strains were clustered together and when compared with 87 global ST398 strains, they were phylogenetically related to a strain identified from China in 2002. The further BEAST analysis (Fig. 1b) showed that all of the ST398 MRSA human isolates from Taiwan shared the common ancestor in 1986 with the human strain isolated from China in 2002 and then were diverged in 2006.

Of noting, five MRSA isolates were identified from five residents in two nursing homes (NHs) in a survey conducted in 2012, and so did for six MRSA isolates from two residents and three health care workers in one NH in a longitudinal survey conducted in 2016 in northern Taiwan. These findings suggest that MRSA ST398 might have been circulating in some NHs recently in Taiwan. In contrast, the phylogeny of the six local ST398 MSSA strains, though all isolated in the same year (2015), was very diverse except for two isolates from a single subject in different time points, which suggest that these isolates might have different origins and might be unrelated to each other (no local transmission). These findings were supported by the BEAST analysis.

There are several limitations of this study. Firstly, since all the ST398 *S. aureus* isolates identified and characterized in this study were only from our research collection, further studies are needed to figure out the whole perspective of ST398 *S. aureus* in Taiwan. Secondly, the nature of present study is retrospective, so in addition to four foreign workers (three from the Philippines and one from Indonesia), the detailed traveling history of going abroad could not be identified exactly from the case patients as well as their household members. Thus, whether the isolates of ST398 from these patients were imported or not cannot be traced clearly.

## Conclusions

Though still uncommon, ST398 *S. aureus* strain was identified in Taiwan since 2012. Among the ST398 *S. aureus* isolates identified in Taiwan, most isolates, particularly MRSA, were human-adapted, though few isolates were potentially livestock-associated. Local transmission of human-adapted MRSA ST398 strains have occurred in some nursing homes in Taiwan after possibly imported from China. Further surveillance of local MRSA molecular epidemiology is needed.

## Data Availability

The data that support the findings of this study are available from the corresponding author upon reasonable request.

## Abbreviations

CA: Community-associated
HCW: Health care worker
IEC: Immune evasion complex
LA: Livestock-associated
MRSA: Methicillin-resistant *Staphylococcus aureus*
NH: Nursing home
PFGE: Pulsed-field gel electrophoresis
PVL: Panton-Valentine leucocidin
SCC: Staphylococcal cassette chromosome
ST: Sequence type
